# Investigating the Co-movement Nexus Between Air Quality, Temperature, and COVID-19 in California: Implications for Public Health

**DOI:** 10.3389/fpubh.2021.815248

**Published:** 2021-12-23

**Authors:** Zeeshan Fareed, Muhammad Farhan Bashir, Bilal, Sultan Salem

**Affiliations:** ^1^School of Economics and Management, Huzhou University, Huzhou, China; ^2^School of Business, Central South University, Changsha, China; ^3^Accounting School, Hubei University of Economics, Wuhan, China; ^4^Department of Economics (DoE), Birmingham Business School (BBS), College of Social Sciences (CoSS), University of Birmingham, Birmingham, United Kingdom

**Keywords:** COVID-19, air quality index, temperature, California, wavelet-analysis

## Abstract

This research aims to look at the link between environmental pollutants and the coronavirus disease (COVID-19) outbreak in California. To illustrate the COVID-19 outbreak, weather, and environmental pollution, we used daily confirmed cases of COVID-19 patients, average daily temperature, and air quality Index, respectively. To evaluate the data from March 1 to May 24, 2020, we used continuous wavelet transform and then applied partial wavelet coherence (PWC), wavelet transform coherence (WTC), and multiple wavelet coherence (MWC). Empirical estimates disclose a significant association between these series at different time-frequency spaces. The COVID-19 outbreak in California and average daily temperature show a negative (out phase) coherence. Similarly, the air quality index and COVID-19 also show a negative association circle during the second week of the observed period. Our findings will serve as policy implications for state and health officials and regulators to combat the COVID-19 outbreak.

## Introduction

In December 2019, coronavirus disease 2019 (COVID-19), a newly discovered infectious coronavirus, was first detected in Wuhan (1–3). According to WHO, COVID-19 can be transmitted from person to person *via* respiratory droplets (4). Later on, after identifying a cluster of COVID-19, the total confirmed cases rose not only in Wuhan but also in the rest of China and turned into an epidemic (5). Initially, Wuhan (6) and later on, the whole country was put on lockdown (7) to ease the health facilities and slow down the transmission of COVID-19 (8). After breakouts of COVID-19 cases in Italy, Iran, and other nations, WHO declared a worldwide health emergency on January 30 (9). Nearly two-thirds of the world's population was placed under some form of lockdown (10). Figure 1 shows the daily COVID19 cases in California state. As we can see from the figure that there is a continued increasing trend throughout the sample period.

**Figure 1:** Daily confirmed new cases of the coronavirus disease 2019 (COVID-19) in California, USA.

Industrial activity came to a halt as the governments gradually enacted lockdown measures. The transportation sector has been struck the hardest since obligatory travel restrictions were put in place to curb the spread of COVID-19 cases (11). According to the aviation industry, COVID-19 has reduced air travel by 96%, the lowest level in the last 75 years (12). Additionally, the demand for fossil fuels drastically declined, and measures were taken to reduce supply as transport, and industrial sectors worldwide came to a halt. COVID-19 has had a negative impact on human health and the global economy, yet the COVID-19 lockdown measures have significantly decreased pollution from economic and commercial activities (5, 13–15). Nitrogen dioxide (NO_2_) is a highly reactive environmental pollutant that is emitted mostly from the industrial and transportation sectors whenever petroleum products (oil and coal) are used (16, 17). According to scientific studies, Nitrogen dioxide is extremely harmful to human health, and it causes respiratory issues, cellular inflammation, and hyperresponsiveness, as well as increasing mortality rates (18). Air pollution has become a major environmental concern, with 4.6 million people dying each year due to poor air quality (19). Moreover, some recent studies suggest that environmental and air quality-related factors have adversely impacted and caused for spreading of COVID-19 cases (20–22). Figure 2 shows the daily average temperature and air quality index in California state.

**Figure 2:** Daily air quality index and the average temperature in California, USA.

### Evaluation of Pollution During COVID-19

The application of lockdown measures to reduce COVID-19 has significantly reduced transportation activities. It has resulted in lower demand for fossil fuels and less energy consumption, which directly impacts environmental quality across the globe. The European Space Agency (ESA) and NASA have released statistical evidence that NO_2_ and other environmental pollutants have been reduced up to 30%, and as a consequence, environmental quality has improved. Satellites images released by ESA and NASA have collected environmental data using the Sentinel-5P satellite and Ozone Monitoring Instruments (OMI) shown in Table 1.

**Table 1:** Assessment of air pollution during the coronavirus disease 2019 (COVID 19).

**Country**	**Time**	**Satellite**	**Agency**	**% Reduction**
China	January and February 2020	Sentinel-5P	ESA	20–30%
Europe	March 2019 and March 2020	Sentinel-5P	ESA	20–30%
Italy	March 2019 and March 2020	Sentinel-5P	ESA	20–30%
France	March 2019 and March 2020	Sentinel-5P	ESA	20–30%
Spain	March 2019 and March 2020	Sentinel-5P	ESA	20–30%
USA	March 2015–19 and March 2020	Aura	NASA	30%

*Source: ESA and NASA*.

Furthermore, Google issued a mobility report for February 23 to April 5, which shows that human mobility in Spain, France, Italy, and USA has been reduced significantly. Human activities are common sources of air pollution, such as power plants, industrial factories, and fossil fuel combustion by airplanes and motor vehicles. These pump air pollutants, such as nitrous oxide, ozone, and carbon monoxide into the earth's atmosphere, contributing to environmental degradation. Table 2 shows the implementation of lockdown measures that have contributed immensely to limiting industrial economies' environmental pollution.

**Table 2:** Mobility index report based on Google tracking.

**Country**	**Residential**	**Transport**	**Parks and outing**	**Retail and recreation**	**Grocery and pharmacy**	**Workplace**	**Parks and outing**
USA	13%	−54%	−20%	−49%	−20%	−40%	−20%
UK	15%	−70%	−29%	−82%	−41%	−54%	−29%
Spain	23%	−89%	−90%	−94%	−77%	−68%	−90%
Germany	8%	−47%	61%	−58%	−13%	−30%	61%
Italy	24%	−86%	−90%	−95%	−82%	−62%	−90%
France	17%	−82%	−73%	−85%	−62%	−53%	−73%

*Source: Google tracking*.

According to the WHO news release, 7 million people die each year due to fine particle exposure in polluted air (23). The Centers for Disease Control and Prevention (CDC) guesstimates that around 360,000 people die every year in the USA alone because of air pollution. The state of California has experienced exponential growth as market reforms introduced to attract investments have made it the USA's economic capital and has improved Californians' living standards, which is evident by the vehicular fleet on the roads in the state. On the contrary, environmental quality has greatly reduced in recent decades. The CDC has listed California to have the worst air quality in the USA as ten^1^ of the top-25 most polluted cities in America are from California.

However, the air quality has greatly improved due to the mandatory lockdown measures adopted by the California state to reduce COVID-19 transmissions (24). California (32°32′N to 42°N, 114°8′W to 124°26′W) is plagued by substantial environmental issues caused by economic activities. It is the world's fifth-largest economy, with a gross domestic product of $3 trillion (larger than France, the UK, and India). To analyze the impact of air pollutants with COVID-19, the data for Air Quality Index (AQI) and COVID-19 cases were taken from the Environmental pollution agency (EPA) and CDC from March 1 to May 25, 2020. The concentration of air pollutants has been compared from January 15 to April 15, 2020, and scientific studies have shown that air pollutants have been reduced up to 60% in California.

## Materials and Methods

Environmental pollution is measured through the AQI, which has been taken from EPA. The daily new confirmed infections representing the COVID-19 outbreak are collected from the official website of CDC. The average daily temperature in California is taken as a proxy for climate indicators and sourced from www.accuweather.com. To examine the correlation between variables, we collected data from March 1 to May 24, 2020. We have employed novel wavelet approaches include “Continuous Wavelet Transform” (CWT), “Wavelet Transform Coherence” (WTC), “Partial Wavelet Coherence” (PWC), and “Multiple Wavelet Coherence” (MWC), to examine the time-varying association between the number of cases reported and the AQI in California. Wavelet methodology is one the most widely used analytical approaches in geosciences, environment, weather, tourism, and economics (25–30). It captures a non-linear association between multiple data series (31). The use of such methodology is also a novelty in the case of COVID-19 and AQI-related studies.

We chose wavelet methodology for current research because of its capacity to handle non-stationary and non-normal data distributions in a time series, which is a huge advantage compared with Fourier analysis. Further, we can study associations in a localized time and at different frequencies. We can measure positive and negative associations at different moments and multiple frequencies in the same graph, which is a unique feature of this technique. Still, another advantage lies in its flexibility to handle different types of distributions with multiple types of wavelet functions available, among which we are using “Morlet wavelet”. The varying wavelet functions allow highly accurate modeling of the association among variables (32–34).

The wavelet transforms coherence is given by Equation 1 as :


(1) $$\begin{array}{l} R^{2}(m,n)=\;\frac{|N(N^{-1}W_{xy}\left(m,n\right)){|}^{2}}{N(N^{-1}|W_{x}(m,n){|}^{2}N(N^{-1}|W_{y}\left(m,n\right)){|}^{2}} \end{array}$$

The wavelet coherence can range from 0 ≤ *R*2 (*m,n*) ≤ 1, where 1 means high coherence and 0 equals no coherence.

### The Partial Wavelet Coherence

In the PWC, we study the coherence between two variables while we control the common effects of the third variable. Equations 2–7 give us the empirical estimations of wavelet coherence.


(2) $$\begin{array}{l} R\left(x_{1},x_{2}\right)=\;\frac{S\left[W\left(x_{1},x_{2}\right)\right]}{\sqrt{S\left[W\left(x_{1}\right)\right]S\left[W\left(x_{2}\right)\right]}} \end{array}$$

(3) $$\begin{array}{l} R^{2}\left(x_{1},x_{2}\right)=R\left(x_{1}x_{2}\right).R{\left(x_{1}x_{2}\right)}^{*} \end{array}$$

(4) $$\begin{array}{l} R\left(x_{1},y\right)=\;\frac{S\left[W\left(x_{1},y\right)\right]}{\sqrt{S\left[W\left(x_{1}\right)\right]S\left[W\left(y\right)\right]}} \end{array}$$

(5) $$\begin{array}{l} R^{2}\left(x_{1},y\right)=R\left(x_{1}y\right).R{\left(x_{1}y\right)}^{*} \end{array}$$

(6) $$\begin{array}{l} R\left(x_{2},y\right)=\;\frac{S\left[W\left(x_{2},y\right)\right]}{\sqrt{S\left[W\left(2\right)\right]S\left[W\left(y\right)\right]}} \end{array}$$

(7) $$\begin{array}{l} R^{2}\left(x_{2},y\right)=R\left(x_{2}y\right).R{\left(x_{2}y\right)}^{*} \end{array}$$

From the above Equations 2 to 7, we can derive the following mathematical expression of partial wavelet coherence;


(8) $$\begin{array}{l} RP^{2}\left(y,x_{1},\;x_{2}\right)=\;\frac{|{R\left(y,x_{1}\right)-R\left(y,x_{2}\right)R\left(y,x_{1}\right)}^{*}{|}^{2}}{{\left[1-R\left(y,x_{2}\right)\right]}^{2}{\left[1-R\left(x_{2},x_{1}\right)\right]}^{2}} \end{array}$$

### The Multiple Wavelet Coherence

The most straightforward approach to comprehend multiple wavelet coherence is to associate it with multiple correlations. This approach allows us to study coherence between dependent variable Y and two independent variables X1 and X2. Equation 9 shows us the numerical representation of the Multiple wavelet coherence.


(9) $$\begin{array}{r} RM^{2}\left(y,x_{2},x_{1}\right)=\\ \frac{R^{2}\left(y,x_{1}\right)+R^{2}\left(y,x_{2}\right)-2R\;e\left[R\left(y,x_{1}\right).R{\left(y,x_{2}\right)}^{*}.R{\left(x_{2},x_{1}\right)}^{*}\right]}{1-R^{2}\left(x_{2},x_{1}\right)} \end{array}$$

## Results and Discussions

Table 3 presents the descriptive statistics highlighting that the average daily cases of COVID-19 is 791.096, with a minimum value “0” to maximum value 2,283. The values for average temperature are 55.33°F, with a minimum value of 43.8°F to a maximum of 74.3°F. The average air quality index value is 42.423 fluctuating between 31 and 61, which shows significant variation during this period. The correlation between COVID-19 and temperature is negative and significant at the 1% level, while the correlation between COVID-19 and AQI is positive at a 1% level of significance. The coefficient value for temperature and COVID-19 is −0.499, the coefficient value for AQI and COVID-19 is 0.241 and the coefficient value for AQI and temperature is 0.572.

**Table 3:** Empirical statistics.

**Variable**	**COVID-19**	**TEMP**	**AQI**
Mean	791.096	55.333	42.423
Std. Dev.	680.157	6.307	6.207
Min	0	43.8	31
Max	2283	74.3	61
Jarque-Bera	7.123	5.251	5.831
*P*	0.028	0.018	0.054
**Correlation matrix**			
COVID-19	1		
TEMP	−0.499^*^	1	
	0.000		
AQI	0.241	0.572*	1
	0.085	0.000	

* *Significant at 1% level*.

Figures 3A–C show continuous wavelet transformation of temperature, AQI, and COVID-19, respectively. A lot of wavelet functions are available for the transformation of time series data. We have used “Morlet wavelet” for this purpose, which suits our data kind and is one of the most extensively used wavelet functions in such transformation recently.

**Figure 3:** Continuous wavelet transform of temperature (TEMP) **(A)**, air quality index (AQI) **(B)**, and COVID-19 **(C)**.

Dark red areas show notable variations, whereas blue areas reveal little variations in respective time-frequency spaces. The only prominent red area in Figure 3A, inside the cone of influence showing such a variation, lies in front of frequency bands 8–16 between the second and third weeks of the observed period, in case of temperature. Figure 3B showing CWT of AQI reveals little variations in frequency space 0–4 and 4–8 during the fourth weeks of the observed period, represented by small red color shapes with black borders inside the so-called cone of influence. COVID-19 varies significantly during the third week of observation in frequency space of 0–4 and 4–8, explained by a large vertical hanging red shape with black borders near the top to Figure 3C.

The results from WTC show us the association between different combinations of pairs of studied variables. The direction of small arrows indicates the causality direction from one variable to the other. The color inside the circles, on the other hand, indicates the strength of a relationship. The strength of the association weakens as we move from red to blue. The Cone of Influence (COI) isolates the significant region with a thick black lining drawn from top to bottom on both sides. The Monte Carlo technique is used to determine the significance level of MWC, WTC, continuous wavelet transform, and PWC. All areas inside the black borders with a red color inside are significant regions.

Figure 4A showing the WTC between temperature and AQI, tells us about a weak relationship between these two variables. At the beginning of the fifth week of observation and in the 4–8 frequency range, the only noteworthy red area with black edges can be noticed. The arrows inside it are rightward directed, telling us a positive coherence. In this case, none of these variables is leading or lagging, as indicated by the “0” degree angle of the arrows. Other red patches can be observed strewn over the diagram, but they don't indicate significant relationships. So, temperature and air quality index are positively related in a specific time–frequency space only.

**Figure 4:** Wavelet Coherence transform of TEMP **(A)**, AQI **(B)** and COVID-19 **(C)**.

Temperature and COVID-19 show a negative relationship from COVID-19 to temperature during the second week of the observed period and in the frequency range of 0–4 time periods, represented by a small red color circle on the top left side of Figure 4B. This implies that an increase in new confirmed cases of COVID-19 leads to a decrease in temperature but only during a short period of time–frequency combination. This impact may be a result of decreased emissions due to lockdown. Figure 4C indicates the wavelet coherence between AQI and COVID19. The WTC of AQI and COVID-19 presents an interestingly negative association running from COVID-19 to AQI represented by the leftward direction of the arrows inside the red circle during the second week of the observed period and frequency area of 4–8 time periods. This implies that COVID-19 leads to a decrease in AQI, tantamount to a better environment. This again may result from low emissions due to reduced industrial, transportation and related activities, a significant source of greenhouse gases.

Figures 5A1,B1,C1 show the PWC results, while Figures 5A2,B2,C2 depict MWC. PWC tells us if the association between two variables remains after canceling the common impact of a third variable. In comparison, MWC reveals the accumulated impact of two independent variables on another third variable as a dependent one. Red areas show a high magnitude of the relationship, while blue areas mean no association. Most of the areas inside Figures 5A1,B1,C1 are blue, indicating only a little or no relationship when we cancel the common effects of COVID-19, temperature, and AQI from the relationship between temperature-AQI, COVID-19-AQI, and temperature-COVID-19, respectively. The association of COVID-19 and temperature still holds as shown by a small red circle on the top left of Figure 5C1. This implies that AQI had no role in the coherence between COVID-19 and temperature, and it is free of the confounding impact of AQI. At the same time, the other two results of WTC, which are altered by the inclusion of a third variable, may not truly represent causation.

**Figure 5:** Partial and multiple wavelet coherence of TEMP, AQI and COVID-19.

COVID-19 and AQI can significantly explain the variation in weather at all frequency ranges except the longest one. This association can be observed during the second to fifth weeks of the observed period, represented by red-colored circles of different sizes scattered inside the cone of influence in Figure 5A2. COVID-19 and AQI had a significant combined impact to explain variations in temperature at specific time-frequency spots during our observed period in California. Figure 5B2 shows how the combined impact of temperature and COVID-19 explains AQI in California through MWC. Multiple red areas in 0–4, 4–8, and 8–16 frequency periods during the third, second and fifth, and fourth week of our observed period exhibit this phenomenon. The air quality seems to be sufficiently explained by the reduced economic activities due to COVID-19 and temperature combined. Temperature and AQI together explain the variations in COVID-19 during the second week of our observation and in the frequency range of 0–4 and 4–8 as shown by red areas in Figure 5C2.

## Conclusion

Air Quality Index (AQI) and climate indicators are critical determinants of the COVID-19 outbreak. AQI and COVID-19 show a negative association circle during the second week of the observed period and frequency area of 4–8 time periods, suggesting that COVID-19 leads to a better AQI, resulting in reduced environmental pollution. This may result from low emissions due to reduced industrial, transportation, and related activities, a significant source of greenhouse gases. Daily temperature and COVID-19 outbreak in California show a negative (in-phase) coherence but only during a short period of time–frequency combination, meaning that temperature played a significant role in limiting COVID-19 though only in the short-term. This result affirms the previous research (7) that temperature may help in containing COVID-19. Although our approach is a relatively better analytical method than correlation and time series methods, as discussed earlier in this study, we should exercise great care in interpreting it as absolute causation. We need a scientific law/theory most of the time. Furthermore, we encourage future research to investigate regional geographical areas as our study is limited to California only.

## Data Availability Statement

The raw data supporting the conclusions of this article will be made available by the authors, without undue reservation.

## Author Contributions

All authors listed have made a substantial, direct, and intellectual contribution to the work and approved it for publication.

## Conflict of Interest

The authors declare that the research was conducted in the absence of any commercial or financial relationships that could be construed as a potential conflict of interest.

## Publisher's Note

All claims expressed in this article are solely those of the authors and do not necessarily represent those of their affiliated organizations, or those of the publisher, the editors and the reviewers. Any product that may be evaluated in this article, or claim that may be made by its manufacturer, is not guaranteed or endorsed by the publisher.

## Footnotes

^1^San Jose, Fresno, Los Angeles, San Diego, Bakersfield, Sacramento, El Centro, Chico, Redding, and Visalia.
